# An Adaptive EEG Classification Algorithm Based on CSSD and ELM_Kernel for Small Training Samples

**DOI:** 10.1155/2022/4509612

**Published:** 2022-12-28

**Authors:** Li Wang, Zhi Lan, Qiang Wang, Xue Bai, Fengling Ma

**Affiliations:** National Research Center for Rehabilitation Technical Aids, No 1 Ronghua Mid-Road, BDA, Beijing, China

## Abstract

Rehabilitation technologies based on brain-computer interface (BCI) have become a promising approach for patients with dyskinesia to regain movement. In BCI experiment, there is often a necessary stage of calibration measurement before the feedback applications. To reduce the time required for initial training, it is of great importance to have a method which can learn to classify electroencephalogram (EEG) signals with a little amount of training data. In this paper, the novel combination of feature extraction and classification algorithm is proposed for classification of EEG signals with a small number of training samples. For feature extraction, the motor imagery EEG signals are pre-processed, and a relative distance criterion is defined to select the optimal combination of channels. Subsequently, common spatial subspace decomposition (CSSD) algorithm and extreme learning machine with kernel (ELM_Kernel) algorithm are used to perform the types of tasks classification of motor imagery EEG signals. Simulation results demonstrate that the proposed method produces a high average classification accuracy of 99.1% on BCI Competition III dataset IVa and 76.92% on BCI Competition IV dataset IIa outperforming state-of-the-art algorithms and obtains a good classification accuracy.

## 1. Introduction

Brain-computer interface (BCI) is a brain-computer communication system that does not depend on the brain's conventional channel. The essence is to identify people's intentions through the electroencephalogram (EEG) signals, so as to realize human-machine communication. BCI has an extensive application prospect in many fields such as rehabilitation engineering, auxiliary control, and entertainment [1–3].

When taking a machine learning approach to BCI, one has to apply labelled training data to teach the classifier. To this end, the user usually performs a necessary stage of calibration measurement before the feedback applications. One important objective in BCI research is to reduce the time required for the initial measurement. Therefore, it is of great importance to have a method that can obtain high classification accuracy with a small number of training samples.

Multichannel EEG signals are usually necessary for spatial pattern identification. Most BCI systems require multichannel EEG data to achieve good performance [4]. However, multichannel EEG data will contain redundant information and noise for data processing and cause inconvenience for practical applications [5–7]. In several cases, there is no clear agreement that exists on the number and location of the necessary channels for motor imagery EEG [8]. Thus, channel selection is necessary for improving the performance of motor imagery-based BCI.

Currently, many feature extraction methods have been widely researched. Not only the characteristics of time-varying, nonstationary, and individuation differences, but also physical state, mood, posture, and other factors pose great difficulties for the analysis of EEG signals. Lin et al. proposed the adaptive autoregressive (AAR) model algorithm [9]. The AAR model parameters can better reflect the changes of event-related EEG signals, but it is sensitive to the artifact. The common spatial pattern (CSP) algorithm of [10] is a classical algorithm toward the analysis of EEG signals. CSP algorithm, however, considers only two types of tasks which have the maximum separability on the projection of space and its performance is affected by nonstationary EEG signals and frequency filtering. Wavelet decomposition (WD) [11] has a lower time resolution and a higher frequency resolution at low frequency and a higher time resolution and a lower frequency resolution at high frequency, which leads to the loss of feature information. Wavelet packet decomposition (WPD) [12] is the development of WD and already has extensive applications [13]. WPD decomposes the low and high frequency information simultaneously in order to improve the time resolution. The coefficients of the wavelet packets include signal information of the frequency bands, but the band-crossing phenomenon exists in every layer of WPD [14]. The classification accuracy may not be high if the band-crossing phenomenon is not considered. Hilbert-Huang Transform (HHT) [15], an adaptive data-driven method, is widely applied for the analysis of nonstationary data. However, the intrinsic mode functions (IMF) criterion for sifting stoppage and boundary extension method of the HHT algorithm will produce some effect on the feature extraction. Common spatial subspace decomposition (CSSD) is an algorithm which is often employed in multichannel EEG data filtering. Each spatial model describes the distribution pattern of specific signals which are located in different regions of the brain. There is a great deal of research value on the synergy work mechanism of multiple brain regions [16]. Regularization factor was introduced based on the CSSD algorithm in [17]. K-nearest neighbor (KNN) algorithm was used to identify motor imagery EEG. The R-CSSD algorithm produced good classification accuracy and less time consumption. In order to relax the presumption of strictly linear patterns between source signals and recorded EEG in CSSD, Gao et al. proposed the kernel CSSD algorithm to extend it to multiclass and obtained better classification results [18]. Grosse-Wentrup et al. proposed a method based on self-adaptive spatial filtering to improve spatial filter using the beamforming technique, and the classification rate was improved [19]. Under small training samples condition, Tomioka and Aihara applied logistic regression with the dual spectral (LRDS) method and obtained good classification accuracy [20]. Park and Lee divided 4–40 Hz band EEG signals into nine sub-bands, and Fisher's Linear Discriminant (FLD) was applied to the features of Regularized CSP (RCSP), which was extracted from individual sub-bands; the proposed method yielded a good classification accuracy in the vicinity of the motor area of the cerebral cortex and obtained particularly excellent performance in small-sample setting situations [21]. Alwasiti et al. proposed the preprocessing pipeline and the triplet network that provide a promising method to classify MI-BCI EEG signals with much less training samples [22]. Singh et al. proposed a new framework that transform covariance matrices into lower dimension through spatial filter regularized by data from other subjects. The efficacy of the proposed approach was validated on the small sample scenario dataset [23]. Hou et al. proposed a novel framework based on bispectrum, entropy, and common spatial pattern (BECSP) for identifying multiclass EEG signals. This algorithm fused features extracted by higher order spectrum, entropy, and CSP algorithm. The tree-based feature selection algorithm was used to select the required features to achieve the purpose of dimensionality reduction and performance improvement [24].

As for classification, SVM [25] has been widely used as a classifier for EEG and has been reported as owning minimum error and producing high classification accuracy, but long time effort needs to be made to find the appropriate parameters for SVM. Other classification techniques are also used such as back-propagation neural network (BP-NN) and KNN. BP-NN is computationally expensive for training and easy to fall into a local optimum. KNN has shown comparable performance with other state-of-the-art methods but its efficiency is greatly reduced when encountering a large amount of training data.

Extreme learning machine (ELM) [26–30] is an algorithm for single-hidden layer feedforward neural networks (SLFNs) with randomly chosen hidden nodes and analytically determined output weights. Since only the output weights between the hidden and output layers are trained, it improves the generalization ability and accelerates the training speed. Gu and Hua proposed a fusion feature that combined temporal and spatial features as the final feature data. The fusion features were input to the trained ELM classifier, and the ELM model achieved a better classification accuracy [31]. Extreme learning machine with kernel (ELM_Kernel) algorithm introduced the kernel function into the ELM algorithm can obtain the minimum square optimization solutions. It solves the problem of random initialization of ELM algorithm, and produces better robustness, better generalization performance, and is more stable with model learning parameters [32].

Thus, as for the aforementioned issue, the combination of ELM_Kernel algorithm and feature extraction based on CSSD algorithm can obtain a good balance between classification accuracy and computational efficiency.

In this paper, the novel combination of feature extraction and classification algorithm is proposed for identification of EEG signals with a small number of training samples. The motor imagery EEG signals are preprocessed, and a relative distance criterion is defined to select the optimal EEG channels. Subsequently, the CSSD algorithm and the ELM_Kernel algorithm are used to classify the types of imagery tasks. Simulation results demonstrate that the channel selection based on the relative distance criterion can enhance the performance of BCI by removing task-irrelevant and redundant channels. The proposed method produces a high average classification accuracy of 99.1% on BCI Competition III dataset IVa and 76.92% on BCI Competition IV dataset IIa outperforming state-of-the-art algorithms and obtains a good accuracy for small training samples. This effectively reduced time consuming of the initial measurement for BCI systems, and helps to pave the way for using BCI systems in the rehabilitation field.

The remainder of this paper is organized as follows: Section 2 specifically analyses the EEG channel selection and the CSSD algorithm.  Section 3 presents the details of ELM_Kernel algorithm.  Section 4 shows the experimental results and analysis.  Section 5 provides the conclusions.

## 2. Feature Extraction

### 2.1. The Acquisition of Experimental Data

The experiment data in this paper comes from BCI Competition III dataset IVa and BCI Competition IV dataset IIa. BCI Competition III dataset IVa poses the challenge of getting along with only a little amount of training data. The recording was made using BrainAmp amplifiers and a 128 channel Ag/AgCl electrode cap from ECI. 118 EEG channels were measured at positions of the extended international 10/20-system. The dataset was recorded from five healthy subjects. Subjects sat in a comfortable chair with arms resting on armrests. Imagery tasks included imagery right hand movement and imagery right foot movement. Given are continuous signals of 118 EEG channels and markers that indicate the time points of 280 cues for each of the 5 subjects (Aa, Al, Av, Aw, and Ay). For some markers no target class information is provided (value NaN) for testing.  Table 1 shows the respective number of training (labelled) trials and test (unlabelled) trials for each subject.

BCI Competition IV dataset IIa [33] consisted of EEG data from 9 subjects (S1–S9). The cue-based BCI paradigm consisted of four different motor imagery tasks. From the four types, we considered only two types, which were imagery left hand movement and imagery right hand movement. EEG signals were recorded and sampled at the rate of 250 Hz using 22 EEG and 3 EOG channels. Only EEG channels were selected for this study. All subjects performed two sessions, one for training and the other for test. The total number of trials per session were 288, with 72 trials per class.

### 2.2. Preprocessing

Event-related desynchronization (ERD) occurs in mu and beta frequency bands, which can be utilized to estimate subject's cognition and emotion states. The raw EEG data is filtered by the band-pass filter with bandwidth of 8–31 Hz in which the ERD physiological feature is apparent.

### 2.3. Channel Selection

The physiological studies on motor imagery demonstrate that the spatial distribution of EEG differs from different imagery movements. EEG oscillations at mu rhythms (8–13 Hz) are displayed on specific areas of ERD corresponding to each imagery state. ERD represents the changes of the ongoing EEG activity characterized by a decrease of power in the given frequency bands. Different degree of ERD is activated via different imagery tasks.

Figure 1 shows the comparison of the AR model power spectrum with 3 randomly selected channels of the imagery right hand and imagery right foot movement on BCI Competition III dataset IVa. The difference in the power spectrum of channel P1 and channel C3 is distinct from the two types of tasks, but the value of the respective power spectrum is not the same. The difference in the power spectrum of channel AF3 is not obvious. It can be distinctly observed that the intensity level of the ERD phenomenon on different channels of the two types of imagery tasks is not the same. In other words, the contribution of different channels to the EEG classification is not the same. It is related to the channel position. Therefore, it gives evidence for channel selection.

Multichannel EEG data applied in BCI systems may contain redundant information and cause inconvenience for practical application. Channel selection can enhance the performance of BCI by removing task-irrelevant and redundant channels. ERD phenomenon produces in specific brain regions. When performing the right hand or right foot imagery movement, only a small amount of channels is activated and some of the channels remain in the stationary state. Therefore, a relative distance criterion is defined to measure the contribution of different channels for identifying tasks so as to select the optimal channels group.

The power spectrum of the two types of imagery tasks is most distinct at 8–13 Hz, which is corresponding to mu rhythm. The relative distance criterion is defined by the difference in the power spectrum between the two types of imagery tasks as follows:

(1) $$\begin{array}{c} h\left(k\right)=\frac{\left|\sum_{f\varepsilon f_{T}}P_{1,k}\left(f\right)-\sum_{f\varepsilon f_{T}}P_{2,k}\left(f\right)\right|}{\left|\sum_{f\varepsilon f_{T}}P_{1,k}\left(f\right)+\sum_{f\varepsilon f_{T}}P_{2,k}\left(f\right)\right|}\text{,} \end{array}$$

where *P*_*i*,*k*_(*f*) denotes the power spectrum density of the *k*-th channel for the *i*-th class, *i*=1 denotes the class of right hand imagery movement, *i*=2 denotes the class of right foot imagery movement, *f* represents frequency, and *f*_*T*_ represents the frequency set of 8–13 Hz.

It can be observed that *h*(*k*) ∈ [0,1], the greater the value of *h*(*k*), the bigger the difference in the power spectrum of the two types of imagery tasks on the same channel and the higher the contribution to classification. The relative distances of all channels are shown in Figure 2. We select the first 25 channels for further analysis that are corresponding to channel F5, FFC3, Fz, F4, CCP3, FC5, FC3, FFC1, FC4, CFC3, CCP5, C3, C1, Cz, C4, CFC4, CCP1, CP3, CPz, CP4, CFC2, P3, Pz, P4, and P8.

### 2.4. Common Spatial Subspace Decomposition Algorithm

CSSD is an algorithm that is often employed in multichannel EEG data filtering. It constructs spatial filters that can distinguish two types of EEG signals based on simultaneous diagonalization of two real symmetric matrices and spatio-temporal source modeling.

Suppose two types of tasks are *A* and *B*. Each subject completes both task *A* and task *B* with the same times, and the time is expressed as *k*. *X*_*A*_ ∈ *R*^*n*×*M*^ and *X*_*B*_ ∈ *R*^*n*×*M*^ denotes two types of tasks EEG by a subject, respectively, *n* denotes the channel number of the EEG signal, *M* denotes sample number of each channel in one trial. So, the feature extraction steps based on the CSSD algorithm are given by the following steps:

**Step 1 .**

Estimate the covariance matrix *R*_*A*_ ∈ *R*^*n*×*n*^ and *R*_*B*_ ∈ *R*^*n*×*n*^ of the two types of imagery EEG signals. The covariance matrix of *A* and *B* for the EEG signal is given by the following equation:

(2) $$\begin{array}{c} \left\{\begin{array}{c} R_{A}=\frac{X_{A}X_{A}^{T}}{\text{trace}\left(X_{A}X_{A}^{T}\right)}\text{,}\\ R_{B}=\frac{X_{B}X_{B}^{T}}{\text{trace}\left(X_{B}X_{B}^{T}\right)}\text{,} \end{array}\right) \end{array}$$

where *X*_*A*_^*T*^ is the transposition of *X*_*A*_, *X*_*B*_^*T*^ is the transposition of *X*_*B*_, and trace(·) is the track of the matrix.

**Step 2 .**

Calculate the sum covariance matrix *R* of the two types of imagery EEG signals and decompose the eigenvalues and eigenvectors, we can obtain the whitening transformation matrix *P* as follows:

(3) $$\begin{array}{c} R=R_{A}+R_{B}=U\cdot \Sigma \cdot U^{T}\text{,}\\ P=\Sigma^{-1/2}\cdot U^{T}\text{,} \end{array}$$

where Σ ∈ *R*^*n*×*n*^ denotes the eigenvalues matrix of *R* and *U* ∈ *R*^*n*×*n*^ is the eigenvectors matrix.

**Step 3 .**

*S*_*A*_ and *S*_*B*_ is obtained from the whitening transformation of *R*_*A*_ and *R*_*B*_ as follows:

(4) $$\begin{array}{c} S_{A}=PR_{A}P^{T}=U_{A}\Sigma_{A}U_{A}^{T}\text{,}\\ S_{B}=PR_{B}P^{T}=U_{B}\Sigma_{B}U_{B}^{T}\text{,} \end{array}$$

where Σ_*A*_ and Σ_*B*_ denotes the eigenvalue matrix, Σ_*A*_+Σ_*B*_=*I*. *U*_*A*_ ∈ *R*^*n*×*n*^ and *U*_*B*_ ∈ *R*^*n*×*n*^ denotes the corresponding eigenvector matrix, *U*_*A*_=*U*_*B*_. For a same eigenvector, if *S*_*A*_ has larger eigenvalues, *S*_*B*_ will have smaller eigenvalues, and vice versa.

**Step 4 .**

Build spatial filter of the two types of imagery EEG signals. Select the biggest *J* eigenvalues from Σ_*A*_ and Σ_*B*_, and we applied the corresponding eigenvectors to form the eigenvector matrix *W*_*A*_, *W*_*B*_ ∈ *R*^*n*×*J*^, the spatial filter of two types of EEG signals is as follows:

(5) $$\begin{array}{c} SF_{A}=W_{A}^{T}P\in R^{J\times n}\text{,}\\ SF_{B}=W_{B}^{T}P\in R^{J\times n}\text{.} \end{array}$$

**Step 5 .**

Suppose *X* ∈ *R*^*n*×*M*^ is the preprocessing EEG signal, the two types of EEG signals are filtered by spatial filter and the feature of EEG is given by the following equation:

(6) $$\begin{array}{c} X_{A}^{a}=SF_{A}\cdot X_{A}\text{,}\\ X_{B}^{b}=SF_{B}\cdot X_{B}\text{.} \end{array}$$

where *v*_*j*_^*A*^ and *v*_*j*_^*B*^ denote the *j*-th (1 ≤ *j* ≤ *J*) row vector of *X*_*A*_^*a*^ and *X*_*B*_^*b*^, respectively.

(7) $$\begin{array}{c} v_{j}^{A^{\prime }}=\log\left[\frac{\text{var}\left(v_{j}^{A}\right)}{\sum_{j=1}^{J}\text{var}\left(v_{j}^{A}\right)}\right]\text{,}\\ v_{j}^{B^{\prime }}=\log\left[\frac{\text{var}\left(v_{j}^{B}\right)}{\sum_{j=1}^{J}\text{var}\left(v_{j}^{B}\right)}\right]\text{.} \end{array}$$

The feature vector of the two types of EEG signals is given by the following equation:

(8) $$\begin{array}{c} V^{A}={\left[v_{1}^{A^{\prime }},v_{2}^{A^{\prime }},\ldots ,v_{j}^{A^{\prime }}\right]}^{T}\text{,}\\ V^{B}={\left[v_{1}^{B^{\prime }},v_{2}^{B^{\prime }},\ldots ,v_{j}^{B^{\prime }}\right]}^{T}\text{.} \end{array}$$

## 3. Classification Algorithm

### 3.1. Basic ELM Algorithm

The ELM algorithm was first proposed by Huang et al. for SLFNs with randomly chosen input weights, hidden nodes, and analytically determined output weights. It possesses an impressive generalization performance.

A standard ELM algorithm classifier is shown in Figure 3, whose *M* hidden nodes use infinitely differentiable activation functions, which could approximate arbitrary samples with zero error, which means given a training set (*x*_*i*_, *T*_*i*_), *i*=1,2,…, *N* where *X*_*i*_=[*x*_*i*1_, *x*_*i*2_,…,*x*_in_]^*T*^ ∈ *R*^*n*^ and *T*_*i*_=[*t*_*i*1_, *t*_*i*2_,…,*t*_im_]^*T*^ ∈ *R*^*m*^, there exist *β*_*j*_, *w*_*i*_, and *b*_*j*_ that make the following equation true.

(9) $$\begin{array}{c} \overset{M}{\underset{j=1}{\sum }}\beta_{j}f\left(w_{i}\cdot X_{i}+b_{j}\right)=o_{i}=T_{i},i=1,2,\ldots ,N, \end{array}$$

where *β*_*j*_ is the weight vector that connects the *j*-th hidden node with the output nodes, *o*_*i*_ is the SLFNs output vector for the *i-*th sample, *T*_*i*_ is the label vector of *i*-th sample, and *w*_*i*_ is the weight vector connecting the *i*-th sample and the *j*-th hidden node, *b*_*j*_ is the bias of the *j*-th hidden node, and *f*(·) is the activation function.

Equation (9) can be replaced by the following equation:

(10) $$\begin{array}{c} H_{w,b,x}\beta =T\text{,}\\ \beta ={\left[\begin{array}{c} \beta_{1}^{T}\\ \vdots \\ \beta_{M}^{T} \end{array}\right]}_{M\times M}\text{,}\\ T={\left[\begin{array}{c} t_{1}^{T}\\ \vdots \\ t_{N}^{T} \end{array}\right]}_{N\times M}\text{,} \end{array}$$

where *H*_*w*,*b*,*x*_ is named the hidden-layer output matrix.

(11) $$\begin{array}{c} H\left(w_{1},\ldots ,w_{M},b_{1},\ldots ,b_{M},x_{1},\ldots ,x_{N}\right)={\left[\begin{array}{ccc} f\left(w_{1}\cdot x_{1}+b_{1}\right) & \cdots & f\left(w_{M}\cdot x_{N}+b_{M}\right)\\ \vdots & \vdots & \vdots \\ f\left(w_{1}\cdot x_{N}+b_{1}\right) & \cdots & f\left(w_{M}\cdot x_{N}+b_{M}\right) \end{array}\right]}_{N\times M}\text{.} \end{array}$$

The smallest training error can be achieved by computing the corresponding least-squares solution *β*=*H*_*w*,*b*,*x*_^†^*T*, where *H*_*w*,*b*,*x*_^†^ is the Moore–Penrose generalized inverse of *H*_*w*,*b*,*x*_.

Altogether, the ELM training algorithm consists of the following three steps:

  Step 1: Randomly assign hidden node parameters *w*_*i*_ and *b*_*j*_, *j*=1,2, ⋯, *N*.
  Step 2: Calculate the hidden-layer output matrix *H*_*w*,*b*,*x*_^†^ and its Moore-Penrose generalized inverse *H*_*w*,*b*,*x*_^†^.
  Step 3: Calculate the output weight *β*.

### 3.2. ELM_Kernel Algorithm

The training process aims to minimize the training error *T* − *Hβ*^2^ and the norm of output weight *β*. The training process can be represented as a constrained optimization problem.

(12) $$\begin{array}{c} \text{Minimize}:\Psi \left(\beta ,\xi \right)=\frac{1}{2}\beta^{2}+\frac{1}{2}C\overset{N}{\underset{i=1}{\sum }}\xi_{i}^{2}\text{,}\\ \text{Subject to}:h\left(x_{i}\right)\beta =t_{i}-\xi_{i},i=1,2,\ldots ,N\text{,} \end{array}$$

where constant *C* is used as a regularization factor to control the tradeoff between the closeness to the training data and the smoothness of the decision function such that generalization performance is improved.

Lagrange multiplier technique is used to solve the above optimization problem. If matrix ((*I*/*C*)+*H*^*T*^*H*) is not singular, solution *β* can be obtained as follows:

(13) $$\begin{array}{c} \beta =H^{T}{\left(I/C+H^{T}H\right)}^{-1}T\text{.} \end{array}$$

Kernel technique can be applied into ELM based on Mercer's condition. Therefore, based on equation (13), the output vector *f*(*x*) of ELM_Kernel can be represented as follows:

(14) $$\begin{array}{c} f\left(x\right)=h\left(x\right)\beta =h\left(x\right)H^{T}{\left(HH^{T}+\frac{I}{C}\right)}^{-1}T\\ ={\left[\begin{array}{c} K\left(x_{i},x_{1}\right)\\ K\left(x_{i},x_{2}\right)\\ \vdots \\ K\left(x_{i},x_{N}\right) \end{array}\right]}^{T}{\left(\frac{I}{C}+K\right)}^{-1}T\text{,} \end{array}$$

where $K=H^{T}H=\left[\begin{array}{ccc} K\left(x_{1},x_{1}\right) & \cdots & K\left(x_{1},x_{N}\right)\\ \vdots & \ddots & \vdots \\ K\left(x_{N},x_{N}\right) & \cdots & K\left(x_{N},x_{N}\right) \end{array}\right]$ and N denotes the number of training samples used for ELM_Kernel.

## 4. Experimental Results and Analysis

The raw EEG signals are large volumes and high dimensionality and will increase the computing time if directly used for classification. Based on the channel selection mentioned in section II, this paper selected 25 channels on BCI Competition III dataset IVa for further analysis.

We apply CSSD algorithm for EEG feature extraction and select the first *J*=10 eigenvalues that are filtered by spatial filter forming the feature vectors. The above feature vectors are brought into the SLFNs, and ELM_Kernel algorithm is applied as the classifying method. This paper sets regularization factor *C* *=* 10, and RBF function is used as the kernel function.

The respective training feature vectors are extracted from the training trials of 5 subjects shown in Table 1. The unlabelled trials are extracted for testing feature vectors, respectively.  Figure 4 shows that the classification accuracy and training time of 5 subjects under BCI Competition III dataset IVa. The proposed algorithm uses an ultrafast time of 0.117 s for training although the subject Al has much more training samples, and the training time is on the decrease as the training samples reduces.

Table 2 summarizes the performance of different combinations of feature extraction and classification methods on BCI Competition III dataset Iva. The ACC represents the average accuracy of EEG and the STD represents the standard deviation. The average classification accuracy of 5 subjects of the proposed algorithm is improved by 2.8% compared with that of the proposed algorithm without channel selection because some channels are irrelevant or redundant. The average classification accuracy of 5 subjects of the proposed algorithm is improved by 4.1% compared with that of the CSSD and ELM algorithm. The reason is that ELM_Kernel algorithm solves the problem of random initialization of ELM algorithm, and produces better robustness, better generalization performance, and is more stable with model learning parameters.

It can be seen from Table 3 that the feature vectors that are extracted based on the CSSD algorithm can effectively characterize EEG signals and the classification accuracy is higher than each item of the results of the 1st BCI Competition and the SBRCSP algorithm on BCI Competition III dataset IVa. The average classification accuracy of 5 subjects of the proposed algorithm is improved by 5% and 16.4% compared with that of the 1st BCI Competition and the SBRCSP algorithm. The high accuracy of the proposed algorithm is depended on the optimal combination of channels and the strong ability of function approximation and better generalization performance of ELM_Kernel algorithm, which is more stable with model learning parameters.

Figure 5 demonstrates that the classification accuracy of different number of eigenvalues that we select based on the CSSD algorithm. It can be observed that 3 eigenvalues poorly characterize the EEG signals, and the classification accuracy is low. The 5 curves own a same trend, the classification accuracy is elevated with the increasing number of eigenvalues. More eigenvalues can effectively characterize EEG signals, but is more time consuming. We obtain great classification accuracy with the first 10 eigenvalues forming the feature vector.

Figure 6 indicates that the classification accuracy of different proportion of the training samples. It can be obviously observed that the proposed algorithm obtains a good accuracy when the proportion of training samples is only 0.1. The accuracy of 5 subjects is different because the EEG signals are affected by physical state, mood, posture, and other factors.

We also compute the classification accuracy with 20 training samples of each subject to further verify the effectiveness of the proposed algorithm under small training samples on BCI Competition III dataset IVa, and the classification accuracy is shown in Table 4. It can be seen that the proposed algorithm obtains higher classification accuracy compared to the BECSP algorithm even though the number of training samples is big. The average classification accuracy of 5 subjects of the proposed algorithm is improved by 11% compared with that of the BECSP algorithm. The high accuracy of the proposed algorithm is depended on the optimal combination of channels and better generalization performance of ELM_Kernel algorithm, which is more stable with model learning parameters. It should be noted that the BECSP algorithm obtains higher classification accuracy compared to the proposed algorithm when the subject is Al. The reason is that the number of training samples of the BECSP algorithm is much more than that of the proposed algorithm.

In order to check for the robustness of the proposed algorithm, we also report the comparison of the proposed algorithm with the BECSP algorithm on BCI Competition IV dataset IIa in Table 5. Simulation result shows that the proposed algorithm can effectively characterize EEG signals and the classification accuracy is higher than each item of the results of the BECSP algorithm. The average classification accuracy of 9 subjects of the proposed algorithm is improved by 5.3% compared with that of the BECSP algorithm.

## 5. Conclusions

In this paper, the novel combination of feature extraction and classification algorithm is proposed based on a little amount of training data for EEG signals using CSSD and ELM_Kernel algorithm. The motor imagery EEG is preprocessed, and a relative distance criterion is defined to select the optimal combination of EEG channels. CSSD algorithm combining with ELM_Kernel algorithm are used to classify the types of imagery tasks. Simulation results demonstrate that the channel selection can enhance the performance of BCI by removing task-irrelevant and redundant channels, the feature vectors can effectively characterize EEG signals and the proposed method produces high classification accuracy and outperforms state-of-the-art algorithms for small training samples. The excellent performance of the classification is obtained as the stable ELM_Kernel algorithm is applied for classification. The advantages of the ELM_Kernel algorithm in terms of both training time and classification accuracy lay a foundation for online classification of EEG. In future studies, the proposed method will be applied to more EEG classification and be further improved and tested so as to make it applicable for clinical applications in the rehabilitation field.

## Figures and Tables

**Figure 1:** Comparison of the power spectrum with different channels. (a) Channel P1. (b) Channel C3. (c) Channel AF3.

**Figure 2:** The contribution of classification on all channels.

**Figure 3:** ELM classifier architecture.

**Figure 4:** Simulation result of 5 subjects.

**Figure 5:** Comparison of the different number of eigenvalues.

**Figure 6:** Comparison of the different proportion of training samples.

**Table 1:** The number of training set and testing set.

	Training (labelled) trials	Test (unlabelled) trials
Aa	168	112
Al	224	56
Av	84	196
Aw	56	224
Ay	28	252

**Table 2:** Comparison of different algorithms (ACC±STD).

	The proposed algorithm	The proposed algorithm without channel selection	CSSD and ELM algorithm
ACC	99.1%±0.09	96.3%±0.29	95.03%±0.21
Aa	96.4%±0.24	94.5%±0.51	94.1%±0.38
Al	100%	100%	100%
Av	100%	91.7%±0.27	90.3%±0.41
Aw	100%	99.6%±0.31	100%
Ay	98.02%±0.2	95.1%±0.36	93.5%±0.26

**Table 3:** Comparison of different algorithms.

	The proposed algorithm (%)	1st BCI competition (%)	SBRCSP algorithm (%)
ACC	99.1	94.17	82.69
Aa	96.4	95.5	86.61
Al	100	100	98.21
Av	100	80.6	63.78
Aw	100	100	89.05
Ay	98.02	97.6	77.78

**Table 4:** Comparison with the BECSP algorithm on BCI competition III dataset IVa.

	The proposed algorithm			BECSP algorithm		
	Training sample	Testing sample	Classification accuracy (%)	Training sample	Testing sample	Classification accuracy (%)
Aa	20	260	88.46	168	112	77.68
Al	20	260	93.84	224	56	100
Av	20	260	100	84	196	73.98
Aw	20	260	99.23	56	224	84.82
Ay	20	260	98.02	28	252	88.1

**Table 5:** Comparison with the BECSP algorithm on BCI competition IV dataset IIa.

	The proposed algorithm (%)	BECSP algorithm (%)
ACC	76.92	71.61
S1	81.08	80.9
S2	66.67	64.24
S3	91.16	85.76
S4	68.75	65.63
S5	51.25	44.79
S6	68.71	54.17
S7	88.29	84.38
S8	90.97	84.03
S9	85.42	80.56

## Data Availability

The data used to support the experiments and the findings of this study are included within the article.
